The article "Medical Image Classification Based on Information Interaction Perception Mechanism" was published in 2021. Journal: Comput Intell Neurosci.

# Medical Image Classification Based on Information Interaction Perception Mechanism

**DOI:** 10.1155/2021/8429899

**Published:** 2021-12-06

**Authors:** Wei Wang, Yihui Hu, Yanhong Luo, Xin Wang

**Affiliations:** ^1^School of Computer and Communication Engineering, Changsha University of Science and Technology, Changsha 410114, China; ^2^Hunan Children's Hospital, Changsha 410000, China

## Abstract

Colorectal cancer originates from adenomatous polyps. Adenomatous polyps start out as benign, but over time they can become malignant and even lead to complications and death which will spread to adherent and surrounding organs over time, such as lymph nodes, liver, or lungs, eventually leading to complications and death. Factors such as operator's experience shortage and visual fatigue will directly affect the diagnostic accuracy of colonoscopy. To relieve the pressure on medical imaging personnel, this paper proposed a network model for colonic polyp detection using colonoscopy images. Considering the unnoticeable surface texture of colonic polyps, this paper designed a channel information interaction perception (CIIP) module. Based on this module, an information interaction perception network (IIP-Net) is proposed. In order to improve the accuracy of classification and reduce the cost of calculation, the network used three classifiers for classification: fully connected (FC) structure, global average pooling fully connected (GAP-FC) structure, and convolution global average pooling (C-GAP) structure. We evaluated the performance of IIP-Net by randomly selecting colonoscopy images from a gastroscopy database. The experimental results showed that the overall accuracy of IIP-NET54-GAP-FC module is 99.59%, and the accuracy of colonic polyp is 99.40%. By contrast, our IIP-NET54-GAP-FC performed extremely well.

## 1. Introduction

Along with a rapid development of artificial intelligence (AI) in the medical industry, its powerful capability in computation and deep learning ability have successfully attracted the attention of medical experts around the world. As an important field of AI medical image recognition application, digestive endoscopy has progressively received more attention as well. The incidence rate of colorectal cancer ranks the third among malignancies in the world [1], and the mortality rate ranks the second [2]. The research shows that the risk of cancer can be greatly reduced if pathological polyps in colon are found and removed in time before cancerization. Therefore, computer-aided diagnosis (CAD) of colonoscopy has always been one of hotspots in AI research.

As artificial intelligence is developing rapidly, the application range of deep convolutional neural networks (CNN) is broadening. CNNs have made huge breakthroughs in image classification [3, 4], semantic segmentation [5], and super-resolution reconstruction [6]. For example, Wang et al. [7] introduced the application and development of CNNs. Benefited from a rapid growth of graphics processing unit, the performance of computer-aided inspection systems has also been further improved. Based on the image classification algorithms using CNNs, the diagnostic efficiency of colonic polyps can be further improved. Wang et al. [8] proposed an improved deep neural network to detect colonic polyp images. The DNN-CAD model constructed by Byrne et al. [9] can output the histological prediction results almost in real time. Mesejo et al. [10] designed and developed a framework that combined machine learning and computer vision algorithms to perform virtual biopsies of proliferative polyps, serrated adenomas, and adenomas. Renner et al. [11] used deep learning combined with transfer learning to train and verify the DNN-CAD model, achieving a high accuracy rate. Komeda et al. [12] designed the CNN-CAD system to identify the nature of polyps in vitro, achieving a high accuracy rate. In 2003, in the experiment of polyp image recognition under white light colonoscopy, the wavelet transform was used as an image classifier for the first time [13, 14]. Since then, various design ideas and innovative techniques were applied to the diagnostic algorithm. Most of the newly proposed network models used public polyp databases [15–18], but the categories and numbers of images in these databases are insufficient. At present, there are three main types of methods for extracting polyp features: handcrafted, end-to-end learning, and hybrid approach [19]. The handcrafted is mainly to obtain the standby boundary information of polyps by using the low-level image processing method and then to define the unique boundary features of polyps with the obtained information. For example, Zhu et al. [20] analyzed the detected boundary curvature. Kang and Doraiswami [21] looked for elliptical shapes associated with polyps. Hwang et al. [22] mainly studied the boundary curvature and related shapes of colonic polyps. The end-to-end learning method uses polyp texture and color information for feature extraction. For example, Gross et al. [23] proposed the use of local binary patterns (LBP). Ribeiro et al. [24] used deep learning methods to detect polyps. The hybrid integrates the advantages of handcrafted and rnd-to-end learning. For example, Tajbakhsh et al. [25] integrated border, texture, and color information to further improve the detection efficiency.

The article "Medical Image Classification Based on Information Interaction Perception Mechanism" was published in 2021. Journal: Comput Intell Neurosci.

The training of CNN needs a large amount of tagged data, but the dataset of pathological images is very scarce. Transfer learning and data enhancement methods can effectively expand the data scale of colon polyp pathological images. The surface texture information of colonic polyps is not obvious, and complex folds on the colon or food residues in the intestinal cavity can be misdiagnosed as colonic polyps. The above factors require higher sensitivity in the detection algorithm. In addition, colonic polyps are of different sizes and their locations are widely distributed. These factors will sabotage the performance of the model and further increase the difficulty of training the model. To solve above problems, this paper designed a channel information interaction perception module (CIIP). Based on this module, an information interaction perception network (IIP-Net) was proposed and verified on the 3-class datasets. On the premise of considering the channel attention mechanism, CIIP combined the attention features of the previous module with the currently extracted attention features. The operation ensures the attention information flows in the feedforward way among the various modules. Compared with other models, the proposed network model significantly improves the accuracy of classification and recognition of colonic polyp images.

## 2. Proposed Network

### 2.1. CIIP Module and IIP-Nets

In CNN, the features extracted by each convolutional layer are different. The shallow convolution layer extracts abstract features such as target edges and colors, and the deep convolution layer extracts specific features such as target contours and shapes. Although deeper networks can extract richer features, there will be problems such as information loss and gradient degradation during feature extraction. Considering the surface texture information of colonic polyps is not obvious, it will lead to model deviation and overfitting, resulting in reduced performance and generalization. Therefore, this paper designed a channel information interaction perception (CIIP) module. Its structure is shown in Figure 1, where “Conv1” and “Conv3” represent 1 × 1 and 3 × 3 convolution layer, respectively. “GAP” represents the global average pooling layer. “FC” represents the linear transformation. “LayerNorm” represents the normalized processing of the layer. “Att1” represents the weight value of the attention channel of the previous module. “Att” represents the weight value of the attention channel of the current module. “ReLU” and “Sigmoid” both represent the activation function. “⊕” represents the feature matrix is added by bit. “⊗” represents the feature matrix is multiplied by bit. “Conv” represents a composite structure including “convolution,” “layer normalization,” and “activation function.”

The article "Medical Image Classification Based on Information Interaction Perception Mechanism" was published in 2021. Journal: Comput Intell Neurosci.

The CIIP module contains convolution kernels of various sizes. In the net, whether the “Att1” exists is judged firstly, which means to determine whether the previous module feeds back the weight value of the attention channel. Then, we select the first branch or the second branch according to the judgment result. The first branch includes a convolutional short connection layer and a global average pooling layer. The second branch includes a convolutional short connection layer, a global average pooling layer, a full connection layer, and a convolutional layer. The function of the convolutional short connection layer of the module is to increase the depth of the network while reducing information loss. The convolution feature map output by the previous convolution module is input into the convolution short connection layer to generate feature map *X*, where  *X* ∈ *R*^*C*×*H*×*W*^. The first “Conv1” is used to reduce the dimensionality and the second “Conv1” is used to increase the dimensionality. The main purpose of this operation is to save calculation time and improve the nonlinear learning ability of the network, without affecting the final model accuracy.

For the first CIIP module, according to the judgment result, the previous module does not obtain the weight value of attention channel “Att1.” The feature map passes through the first branch. Firstly, the convolution feature map output by the previous convolution module is input into the convolutional short connection layer of the CIIP module to obtain the feature map *X*. Secondly, the feature map *X* is input into the GAP layer. Then, the resulting pooling feature is activated through Sigmoid. Finally, the “Output” is made up of two parts:

(1) The output of the convolutional short connection layer and the attention map are multiplied by bits, and the output features obtained can be expressed as
  (1) $$\begin{array}{c} X^{\prime }=S\left[\text{GAP}\left(X\right)\right]⊗X. \end{array}$$
(2) The feature extracted through the GAP layer and the attention map is multiplied by bits, and the attention channel weight value obtained can be expressed as
  (2) $$\begin{array}{c} \mathrm{Att}=S\left[\text{GAP}\left(X\right)\right]⊗\text{GAP}\left(X\right). \end{array}$$

For the second and third CIIP modules, according to the judgment result, the forward feedback of the previous module has obtained the attention channel weight value “Att1.” The feature map passes through the second branch. First, for the feature map *X* generated by the convolutional short connection layer, pass it through a GAP layer to obtain pooling feature. For the attention channel weight value “Att1” obtained by the feedback of the previous module, pass it through a FC layer (followed by the “LayerNorm” and “ReLU”) to match the channel size. Then, the pooling feature that integrates the global spatial information and the attention channel weight value through channel adaptive matching are stitched bitwise to obtain the convolutional feature. Then, pass it through the “conv” and “sigmoid.” Finally, the “Output” is made up of two parts:

(1) The output of the convolutional short connection layer and the attention map are multiplied by bits, and the output features obtained can be expressed as
  (3) $$\begin{array}{c} X^{\prime }=S\left\{\mathrm{Conv}\left[\left[\delta \left[\text{LN}\left[\ell \left(\mathrm{Att}\right)\right]\left(\right]\right]\left(\right]\left(\right]⊕\text{GAP}\left(X\right)\right]\right]\left(\right]\right\}⊗X. \end{array}$$
(2) The feature extracted through the GAP layer and the attention map is multiplied by bits, and the attention channel weight value obtained can be expressed as
  (4) $$\begin{array}{c} \text{Att}=S\left\{\mathrm{Conv}\left[\left[\delta \left[\text{LN}\left[\ell \left(\text{Att}1\right)\right]\right]⊕\text{GAP}\left(X\right)\right]\right]\right\}⊗\text{GAP}\left(X\right), \end{array}$$

where “*ℓ*” stands for “FC” linear transformation, “LN” means “LayerNorm” layer normalization processing, “*δ*” stands for the “ReLU” activation function, and “*S*” stands for the “Sigmoid” activation function.

The article "Medical Image Classification Based on Information Interaction Perception Mechanism" was published in 2021. Journal: Comput Intell Neurosci.

In this way, the previous module features and the currently extracted features are merged. The operation ensures that the information flows in a feedforward way between each module, and we enhance the feature extraction ability of the network. This is shown in Figure 2.

Based on the CIIP module, this paper proposed a convolutional neural network structure with three depths: information interaction perception network (IIP-Net) 54, IIP-Net105, and IIP-Net156. Due to the different selection of branches, the number of layers of the CIIP structure is also different. The first CIIP structure has three layers, and the second and third CIIP structures have five layers. “Conv” is represented as a composite structure including “convolution,” “batch normalization,” and “activation function.” The network structure is shown in Table 1.

For image classification and for image classification problems, the classifiers of classic networks such as AlexNet and VGGNets are all three-layer fully connected layers. The three-layer fully connected layer has a huge amount of parameters, which increases the calculation time and cost. Moreover, these networks are prone to overfitting, resulting in low generalization ability. Therefore, the single-layer fully connected layer “FC” is used as the classifier in this paper. This is shown in Figure 3(a).

The article "Medical Image Classification Based on Information Interaction Perception Mechanism" was published in 2021. Journal: Comput Intell Neurosci.

This paper introduces the global average pooling (GAP) method proposed by Lin et al. [26]. Different from traditional full connection layers, GAP layers can accept images of any size. First, an average value is calculated for all pixels of the output feature map of each channel. Then, the average value is input to a global average pooling layer, a feature vector of one dimension is obtained, and finally the feature vector is directly input to the softmax layer. In this way, on the one hand, the number of parameters can be reduced to prevent overfitting, and on the other hand, it integrates global spatial information and achieves better robustness. This paper introduces a “GAP-FC” structure, which is composed of GAP and FC. First, the output feature map of the last convolutional layer is reduced to 1 × 1 through GAP, and then, we classify it through a full connection layer. The operation greatly reduces the number of network parameters. The GAP-FC structure is shown in Figure 3(b).

GAP actually calculates the average value of all pixels for each feature map and outputs a data value. Therefore, this paper introduces a “C-GAP” structure, which is composed of point convolution and GAP. First, a 1 × 1 point convolutional layer is used to reduce the dimensionality of the output feature, and then, through the GAP layer, finally, a Softmax function is connected for classification. In this way, the classifier does not include a fully connected layer, further reducing the number of parameters. Compared with “C-GAP” module, the “GAP-FC” module has a larger amount of parameters, but its calculation amount is less than that of “C-GAP” module. The structure of “C-GAP” is shown in Figure 3(c).

### 2.2. Network Complexity

When using different classifiers and different depths' networks to recognize colonic polyp images, the number of parameters and calculations are different. Taking the 3-class classification task as an example, we suppose the size of the output feature map of the last layer of the network is *H* × *W* × *D*. When using the “FC” as the classifier, the number of parameters in the classifier is  *H* × *W* × *D* × 3+3. When using the “GAP-FC” as the classifier, the number of parameters in the classifier is  *D*+*D* × 3+3. When using the “C-GAP” as the classifier, the number of parameters in the classifier is *H* × *W* × 3+*D* × 3+3.

The number of IIP-Net parameters of different depths with different classifiers is shown in Figure 4, and the amount of calculation of different networks is shown in Figure 5.

The article "Medical Image Classification Based on Information Interaction Perception Mechanism" was published in 2021. Journal: Comput Intell Neurosci.

As can be seen from Figure 4, different classifiers will cause huge differences in the amount of network parameters. When the depth of IIP-Net is the same, network parameters using “FC” as a classifier are about 10 million more than network parameters which use other classifiers. Therefore, in the same experimental environment and limited computational memory, when ensuring the accuracy, the use of “FC” as the classifier should be avoided as much as possible. In addition, the number of parameters of IIP-NET156-FC is 1.04 times that of IIP-NET105-FC, and the number of parameters of IIP-NET105-FC is 1.06 times that of IIP-NET54-FC. It can be seen that when the same classifier is used, the network depth also has a great influence on the number of network parameters.

It can be seen from Figure 5 that network depth is the main factor influencing the amount of calculation. The calculation amount of IIP-Net156-FC is 1.46 times that of IIP-Net105-FC. The calculation amount of IIP-Net105-FC is 1.86 times that of IIP-Net54-FC. The calculation amount of IIP-Net156-FC is 2.72 times that of IIP-Net54-FC. With the increase of network depth, the amount of calculation increases sharply. Therefore, in the same experimental environment, the IIP-Net105 model has the highest cost performance when the model accuracy gap is not large.

In summary, by comparing the parameters and calculations number of the network combining three different classifiers, it can be found that the number of parameters using “GAP-FC” and “C-GAP” is about 10 million less than the number of parameters using “FC,” and the number of calculations using “GAP-FC” is about 200 million less than the number of calculations using “GAP-FC” and “FC.” Therefore, under the premise of guaranteed accuracy, “GAP-FC” is the optimal classifier.

## 3. Experimental Results

### 3.1. Preprocessing and Dataset

At present, the number of datasets related to colonic polyps and the number of pictures contained in these datasets are both small. Therefore, our laboratory randomly selected colonoscopy images taken by the olympus PCF-H290DI equipment from the gastrointestinal endoscopy database. Before labeling, the images were cropped to remove the white borders around them, and the size of the images was unified to 256 × 256. After the relevant physicians review the images, then we labeled them; a dataset Dataset-A containing 22809 images is constructed. The dataset includes 4002 colonic polyp images, 14,801 normal images, and 4006 images of other lesions such as colitis.

In the training experiment, the training set consisted of 3002 images randomly selected from 4002 colon polyp images, 11001 images randomly selected from 14801 normal images, and 3006 images randomly selected from 4006 other lesion images. Train the parameters of the model through multiple experiments. Then, the remaining 1000 polyp images, 3800 normal images, and 1000 other lesion images form a test set to verify the performance of the model. In the nonpolyposis dataset, there are not only pictures of colon without lesions but also pictures of colon lesions other than polyps, such as adenomas and inflammatory polyps. For most polyp pictures, polyps do not completely appear in the field of vision; some polyps even only appear in the corners of the picture. In addition to the influence of light, shooting angle, etc., these increase the recognition difficulty. Therefore, we expanded the training set and test set images, including random horizontal flip, random vertical flip, random rotation a certain angle between +90° and −90°, brightness, and contrast changes. These operations greatly increase the amount of data. In fact, the total number of image samples involved in the experiment is 5 times of the original data, reaches 114,045. Data enhancement not only increases the number of samples but also enhances the generalization ability of the model.

The article "Medical Image Classification Based on Information Interaction Perception Mechanism" was published in 2021. Journal: Comput Intell Neurosci.

In order to further verify the generalization performance of CIIP-Net, based on Dataset-A of three categories, a four-category dataset Dataset-B containing 10660 images is constructed. The four categories are colonic polyps, ulcerative colitis, normal, and other lesions. The training set consisted of 9693 images, including 2000 colonic polyp images, 693 ulcerative colitis images, 5000 normal images, and 2000 other lesions images. The test set consisted of 967 images, including 200 colonic polyp images, 70 ulcerative colitis images, 500 normal images, and 197 other lesions images. The vegetation growing on the surface of human mucosa is generally referred to as polyps, so obvious protrusions can be seen in the picture of colonic polyps. Ulcerative colitis refers to ulcerative lesions in the intestinal mucosa, so unevenly distributed ulcers can be seen in the picture of ulcerative colitis. Other lesions include chronic specific colitis and amoebic bowel disease. Different pathological pictures have different characteristics. The images are shown in Figure 6.

### 3.2. Experiment Setup

The experiments in this paper are carried out on the same platform and environment to ensure the credibility of comparisons between different network models. Experiments are conducted on Windows 10 with Intel i7 3.30 GHz CPU, GeForce GTX 1080Ti (11G) GPU, CUDNN 10.0, CUDA 10.0, and CUDA 10.0. The framework is Pytorch. The development tool is PyCharm. The language is Python. The “BatchSize” of the training set and the test set are both set to 32. The learning rate is 0.001. The weight attenuation is 5*E* − 4. The momentum is 0.9. The training period is 100 epochs.

The article "Medical Image Classification Based on Information Interaction Perception Mechanism" was published in 2021. Journal: Comput Intell Neurosci.

### 3.3. Evaluation Criteria

Based on the evaluation criteria adopted by most medical image classification models, this paper used accuracy, precision, recall, F1-measure, and specificity as performance indicators.

The polyp samples are set as positive samples, and the remaining are set as negative samples. The negative samples include normal samples and nonpolyposis samples. TP refers to the number of pixels belonging to the polyp and is correctly classified. FP refers to the number of pixels belonging to the nonpolyposis but wrongly classified as polyps. FN refers to the number of pixels belonging to the polyp but wrongly classified as nonpolyposis. TN refers to the number of pixels belonging to the nonpolyposis and correctly classified as polyps. Evaluation parameters are

(5) $$\begin{array}{c} \;\mathrm{Accuracy}=\frac{\mathrm{TP+TN}}{\mathrm{TP+TN+FP+FN}},\\ \mathrm{Precision}=\frac{\mathrm{TP}}{\mathrm{TP+FP}},\\ \mathrm{Recall}=\frac{\mathrm{TP}}{\mathrm{TP+FN}},\\ F1-\mathrm{Measure}=2*\frac{\mathrm{Recall*Precision}}{\mathrm{Recall+Precision}},\\ \mathrm{Specificity}\frac{\mathrm{TN}}{\mathrm{TN+FP}}. \end{array}$$

The confusion matrix is shown in Table 2.

### 3.4. Experimental Results

In order to study the effect of the depth and classifier of IIP-NET on the colonic polyp images classification performance, 9 types of IIP-NET have carried out classification experiments on colonic polyp datasets with three categories. The experimental results are shown in Table 3. The optimal experimental results are bolded.

According to Table 3, the performance of the model using GAP-FC as the classifier is obviously better. The overall performance of IIP-NET54-GAP-FC is the best, and its accuracy, precision, recall, *F*1-measure, and specificity are all the highest values in the table, which are 99.59%, 99.40%, 99.40%, 99.70%, and 99.40%, respectively, but its classification accuracy of colonic polyps is slightly lower. The accuracy of colonic polyps of IIP-Net105-GAP-FC and IIP-Net158-GAP-FC is the same as 99.50%, and the overall accuracy is also the same as 99.55%. Compared with IIP-Net54-GAP-FC, although the overall accuracy of IIP-Net105-GAP-FC and IIP-Net158-GAP-FC is lower, the gap is very small. The phenomenon indicates that, with the deepening of the network, the network performance does not change significantly. The calculation amount of IIP-Net156 is 1.06 times that of IIP-Net105 and 1.15 times that of IIP-Net54. The parameter amount of IIP-Net156 is 1.47 times that of IIP-Net105 and 2.81 times that of IIP-Net54. After comprehensive consideration, t IIP-NET54-GAP-FC is selected as the recommended model. The three categories confusion matrix of IIP-Net54-GAP-FC is shown in Figure 7.  Table 4 gives more detailed results on the three categories recognition performance of IIP-Net54-GAP-FC.

The article "Medical Image Classification Based on Information Interaction Perception Mechanism" was published in 2021. Journal: Comput Intell Neurosci.

According to Table 4, IIP-Net50-GAP-FC has a good classification performance for polyp images of colonic polyp positive patients, normal patients, and other colonic disease patients. Especially, the classification accuracy, recall, and specificity of colonic polyps are as high as 99%.

We further compare the experimental results of IIP-Net54-GAP-FC with traditional CNNs ResNet50, VGG16, DenseNet121, and GoogLeNet. The experimental results are shown in Table 5, and the optimal experimental results are shown in bold.

ResNet50 solves problems of network degradation and gradient explosion with the deepening of network depth by using skip connections, but the accuracy rate is the lowest in the comparison experiment, only 97.07%. The accuracy rate of VGG16 is about 2.5% lower than that of IIP-Net54-GAP-FC because of its shallow network depth and insufficient image feature extraction, resulting in low image classification accuracy. Moreover, VGG16 uses a three-layer fully connected layer as a classifier, and the amount of parameters and calculations are very large, which greatly increase the calculation time and cost. DenseNet121 realizes the reuse of features by introducing dense connections and further deepens the network depth. Although DenseNet121 achieves good classification accuracy on colonic polyp images, its accuracy is still lower than IIP-Net54-GAP-FC. DenseNet121 also uses a three-layer fully connected layer as a classifier, which makes the amount of calculation and parameter increase dramatically. GoogLeNet achieves good accuracy on colonic polyp datasets, but its performance indicators are all lower than IIP-Net54-GAP-FC. The CIIP module can merge the previous module features with the current extracted features, which further improves the learning ability of the module.

We further compare IIP-Net50-GAP-FC with the methods proposed by Tan et al. [31], Han et al. [32], Wang et al. [9], etc. These methods have achieved good accuracy in colonic polyp classification experiments. The results are shown in Table 6. The optimal experimental results are bolded.

GhostNet has achieved good accuracy on colonoscopy image datasets, but its performance indicators are all lower than IIP-Net54-GAP-FC. Although the overall accuracy rate of VGG19-GAP is up to 98.93%, its accuracy for colonic polyp is only 87.90%, so the clinical utility of this network is not strong. The overall accuracy of other methods is generally lower than the IIP-Net54-GAP-FC. According to Table 6, the overall accuracy and the colonic polyp classification accuracy of the proposed IIP-Net have reached a very high level, which shows that IIP-Net54-GAP-FC performance is better and more targeted for colonic polyp image classification tasks.

The article "Medical Image Classification Based on Information Interaction Perception Mechanism" was published in 2021. Journal: Comput Intell Neurosci.

We use the IIP-Net54-GAP-FC model to perform classification experiments on the Dataset-B with four categories, which improves the difficulty of the classification and recognition task and further verifies the generalization ability of the model in colonoscopy images classification and recognition tasks. The “BatchSize” of the training set and the test set are both set to 16. The learning rate is 0.001. The weight attenuation is 5*e* − 4. The momentum is 0.9. And the training period is 200 epochs.  Figure 8 shows the four categories confusion matrix of IIP-Net54-GAP-FC.  Table 7 gives more detailed results for the four categories recognition performance of IIP-Net54-GAP-FC.

According to Table 7, IIP-Net54-GAP-FC has good classification performance on colonoscopy images of colonic polyp positive patients, ulcerative colitis patients, normal patients, and other colonic disease patients. Especially, the classification accuracy, recall, and specificity of colon polyp are as high as 100%.

We further compare IIP-Net50-GAP-FC with the methods proposed by Tan et al. [31], Han et al. [32], Wang et al. [9], etc. The results are shown in Table 8. The optimal experimental results are shown in bold.

According to Table 8, in the four categories experiment of colonic polyps, the overall accuracies of other methods have reached more than 90%, but the accuracy of colonic polyp is low. Although the overall accuracy of VGG19-GAP is up to 95.35%, its accuracy for colonic polyp is only 88.32%, which is 11.68% lower than IIP-Net54-GAP-FC. In summary, the proposed IIP-Net54-GAP-FC is better, and it has excellent performance in colonic polyp image classification experiments.

### 3.5. Experiments' Analysis

According to the experimental results, in the three categories experiments of colonoscopy images, IIP-Net54-GAP-FC has the highest overall recognition accuracy (99.59%). Although the classification accuracy of colonic polyp is slightly higher (99.40%), it is comparable to IIP-Net105-GAP-FC; IIP-Net158-GAP-FC only differs by 0.1%, and the number of parameters and calculations of network classifier are reduced. In order to further evaluate the generalization ability of the model, IIP-Net54-GAP-FC conducted experiments on the four-category dataset. Comparing the above experimental results with other methods, the overall accuracy and the classification accuracy of colonic polyp are 96.59% and 100%, respectively. The overall performance is better than other methods.

The article "Medical Image Classification Based on Information Interaction Perception Mechanism" was published in 2021. Journal: Comput Intell Neurosci.

Through experimental analysis, it can be seen that, in the colonoscopy images' classification task, the network depth should be kept moderate. If the network is too shallow, it is difficult to fully extract the features. Although deepening the network can make the model have better nonlinear expression ability, deep networks will cause problems such as gradient instability and network degradation. Batch normalization can effectively solve the instability problems such as gradient dispersion and explosion. The convolutional short connection layer can effectively solve the problem of network degradation. The introduction of GAP into the classifier can effectively reduce the amount of network parameters and calculations. The surface texture information of colonic polyps is not obvious; it will lead to model deviation and overfitting, resulting in reduced performance and generalization. Therefore, this paper designed a CIIP module consists of two branches. In the module, whether the previous module has generated the attention channel weight value is judged firstly, and then, different branches are selected according to the judgment result. The first branch contains Conv1, Conv3, and GAP structures. The second branch contains Conv1, Conv3, GAP, and FC structures. Conv1 is used to control the dimension and reduce the number of parameters. Short connections are used to prevent information loss, increase network depth, and solve the problem of network degradation to a certain extent. The input feature map is input to the CIIP module. Because the module can merge the previous module features with the current extracted features, it ensures the information flow in the feedforward way among the modules and enhances the feature extraction ability of the network.

## 4. Conclusions

This paper designed a CIIP module based on the characteristics of colonic polyp images and proposed an IIP-Net to classify colonic images. Colonoscopy images were selected to annotate two colonic polyp image datasets: three-category dataset Dataset-A and four-category dataset Dataset-B. Analyzing and comparing the experimental results, IIP-Net54-GAP-FC has the highest application value.The overall accuracy of the three-category experiment and colonic polyp category accuracy have reached 99.59% and 99.40%, respectively. The overall accuracy of the four-category experiment and colonic polyp category accuracy have reached 96.59% and 100%, respectively. IIP-Net has extremely high accuracy and recall for colonic polyp cases and can effectively help medical imaging physicians detect colonic polyp cases. Despite the good results, IIP-Net still needs clinical research and testing. Moreover, the colonoscopy image datasets' collection and processing process is very difficult. Not only children's colonic polyp image data but also more colonic polyp image data of different ages can be obtained. Through these enhanced image data, the accuracy of CIIP-net can be further improved.

The article "Medical Image Classification Based on Information Interaction Perception Mechanism" was published in 2021. Journal: Comput Intell Neurosci.

## Figures and Tables

**Figure 1:** The structure of CIIP module.

**Figure 2:** The diagram of forward feedback.

**Figure 3:** The structure of the classifier. (a) FC structure, (b) GAP-FC structure, and (c) C-GAP structure.

**Figure 4:** The parameters comparison of IIP-Net.

**Figure 5:** Comparison of floating points of operations (FLOPs).

**Figure 6:** Images in Dataset-B: (a) colonic polyps, (b) ulcerative colitis, (c) other lesions, and (d) normal pictures.

**Figure 7:** Three categories confusion matrix of IIP-Net50-GAP-FC.

**Figure 8:** Four-category confusion matrix of IIP-Net54-GAP-FC.

**Table 1:** The structure of IIP-Net.

Conv7-64, stride:2					
3 × 3Maxpool, stride:2					
Conv1-64	**×**2	Conv1-64	**×**2	Conv1-64	**×**2
Conv3-64		Conv3-64		Conv3-64	
Conv1-256		Conv1-256		Conv1-256	

**CIIP-256**					
Conv1-128	**×**3	Conv1-128	**×**3	Conv1-128	**×**7
Conv3-128		Conv3-128		Conv3-128	
Conv1-512		Conv1-512		Conv1-512	

**CIIP-512**					
Conv1-256	**×**5	Conv1-256	**×**22	Conv1-256	**×**35
Conv3-256		Conv3-256		Conv3-256	
Conv1-1024		Conv1-1024		Conv1-1024	

**CIIP-1024**					
Conv1-512	**×**3	Conv1-512	**×**3	Conv1-512	**×**3
Conv3-512		Conv3-512		Conv3-512	
Conv1-2048		Conv1-2048		Conv1-2048	

**GAP-FC**					
**Softmax**					

**Table 2:** Confusion matrix.

Confusion matrix		Actual class	
		Positive sample (polyp)	Negative sample (nonpolyp)
Predicted class	Positive sample (polyp)	TP	FP
	Negative sample (nonpolyp)	FN	TN

**Table 3:** Performance of different depth IIP-Net (%).

Model	Accuracy	Precision	Recall	Specificity	*F*1-measure	Polyp Acc
IIP-Net54-GAP-FC	**99.59**	**99.40**	**99.40**	**99.70**	**99.40**	99.40
IIP-Net54-FC	94.98	94.88	94.60	98.94	94.74	94.20
IIP-Net54-C-GAP	95.48	96.68	96.10	99.31	96.39	95.90
IIP-Net105-GAP-FC	99.55	99.31	99.31	99.65	99.31	**99.50**
IIP-Net105-FC	95.24	97.24	95.00	99.44	96.11	94.30
IIP-Net105-C-GAP	95.98	97.25	95.40	99.44	96.32	95.40
IIP-Net156-GAP-FC	99.55	99.28	99.28	99.64	99.28	**99.50**
IIP-Net156-FC	93.81	92.34	94.00	98.38	93.16	94.40
IIP-Net156-C-GAP	95.28	97.25	93.80	99.13	95.49	94.40

**Table 4:** Accuracy, recall, and specificity of 3-class IIP-Net54-GAP-FC (%).

Class	Accuracy	Recall	Specificity
Polyp	99.40	99.40	99.87
Normal	99.79	99.79	99.60
Others	99.00	99.00	99.62
Average	99.40	99.40	99.70

The article "Medical Image Classification Based on Information Interaction Perception Mechanism" was published in 2021. Journal: Comput Intell Neurosci.

**Table 5:** Performance of other CNNs (%).

Model	Accuracy	Precision	Recall	Specificity	*F*1-measure	Polyp Acc
ResNet50 [27]	97.07	95.84	95.66	97.83	95.65	98.40
VGG16 [28]	97.08	95.33	95.11	97.55	95.09	96.30
DenseNet121 [29]	97.26	96.22	96.15	98.07	96.15	97.10
GoogleNet [30]	98.26	97.34	97.30	98.65	97.29	98.50
IIP-Net54-GAP-FC	**99.59**	**99.40**	**99.40**	**99.70**	**99.40**	**99.40**

**Table 6:** Comparison of the proposed method with other existing deep learning method.

Name	Class	Method	Accuracy	Polyp Acc
Tan et al. [31]	3	MnasNet0_5	94.57	94.30
Han et al. [32]	3	GhostNet	98.07	97.00
Wang et al. [8]	3	VGG19-GAP	98.93	97.10
Wang et al. [8]	3	ResNet101-GAP	96.43	87.90
Proposed method	3	IIP-Net54-GAP-FC	**99.59**	**99.40**

**Table 7:** Accuracy, recall, and specificity of 4 class IIP-Net54-GAP-FC (%).

Class	Accuracy	Recall	Specificity
Polyp	100	100	100
Normal	98.60	98.60	98.14
Others	88.83	88.83	95.25
Ulcerative colitis	87.14	93.64	97.88
Average	93.64	95.27	97.82

**Table 8:** Accuracy comparison of our proposed method with other existing deep learning method.

Name	Class	Method	Accuracy	Polyp Acc
Tan et al. [31]	4	MnasNet0_5	91.93	78.17
Han et al. [32]	4	GhostNet	93.18	79.70
Wang et al. [8]	4	VGG19-GAP	95.35	88.32
Wang et al. [8]	4	ResNet101-GAP	93.38	86.29
Proposed method	4	IIP-Net54-GAP-FC	**96.59**	**100**

## Data Availability

The dataset can be obtained from the corresponding author upon request.
